The article "Evaluation of the Antiulcer Activity of Methanolic Extract and Solvent Fractions of the Leaves of Calpurnia aurea (Ait.) Benth. (Fabaceae) in Rats" was published in 2022. Journal: Evid Based Complement Alternat Med.

# Evaluation of the Antiulcer Activity of Methanolic Extract and Solvent Fractions of the Leaves of *Calpurnia aurea* (Ait.) Benth. (Fabaceae) in Rats

**DOI:** 10.1155/2022/4199284

**Published:** 2022-06-29

**Authors:** Yared Andargie, Woretaw Sisay, Mulugeta Molla, Alefe Norahun, Pradeep Singh

**Affiliations:** ^1^School of Pharmacy, College of Medicine and Health Science, Debre Tabor University, Debre Tabor, Ethiopia; ^2^Department of Pharmacy, Teda Health Science College, Gondar, Ethiopia

## Abstract

**Introduction:**

In Ethiopia, traditionally, the leaves of *Calpurnia aurea* have been utilized to treat peptic ulcer disease. Therefore, the objective of the present study was to examine the antiulcer activity of *Calpurnia aurea* hydromethanolic leaf extract and solvent fractions in rats.

**Methods:**

The ulcer-healing potential of the crude test extract was assessed in rats by adopting pyloric ligation-, acidified ethanol-, and acetic acid-induced ulcer methods; while, in solvent fractions, the acidified ethanol-induced ulcer model was used. In all models, three serial test doses (100, 200, and 400 mg/kg) were given and the antiulcer activity was investigated. Standard drugs like sucralfate (100 mg/kg), omeprazole (20 mg/kg), and cimetidine (100 mg/kg) have been used as a positive control; whereas distilled water (10 mL/kg) was used as the negative control. Parameters like ulcer index, total acidity, pH, gastric volume, and gastric mucin level were all measured.

**Results:**

In an acute toxicity study, the test extract at the limit test dose (2 g/kg) was safe following a single dose administration. In pyloric ligation-induced ulcers, the plant extract at 200 and 400 mg/kg significantly reduced the ulcer index, the volume of stomach secretion, and total acidity while raising gastric pH and mucus content (*P* < 0.05). Likewise, in the acidified ethanol- and acetic acid-induced ulcer models, the extract at both test doses (200 and 400 mg/kg) also displayed a substantial reduction (*P* < 0.05) in ulcer index. Among the fractions, the ethyl acetate fraction revealed remarkable cytoprotective activity at all test doses and the aqueous fraction at 400 mg/kg (*P* < 0.05). In contrast, the effect of chloroform fraction was found to be negligible. The peak ulcer inhibition was noted at 400 mg/kg of ethyl acetate fraction (52.4%).

**Conclusion:**

The study showed that the crude extract and solvent fractions possess remarkable antiulcer activity.

## 1. Introduction

Peptic ulcer disease is characterized by painful sores or lesions in the stomach wall or the first portion of the small intestine, known as the duodenum. It is also termed as peptic ulcer or gastric ulcer, which is a breach in the gastric wall or, some instances, in the lower portions of the esophagus [1]. It is a recurrent and persistent condition manifested by right upper quadrant pain. Epidemiological studies indicated that peptic ulcer is the most frequent gastrointestinal malady globally, with high fatality rates [2]. The disorder is widespread worldwide, with annual incidences ranging from 0.10% to 0.19% for physicians and 0.03% to 0.17% for hospital-diagnosed peptic ulcers [3]. It is caused by a high accumulation of offensive factors and a lack of protective factors in the stomach [4].

The article "Evaluation of the Antiulcer Activity of Methanolic Extract and Solvent Fractions of the Leaves of Calpurnia aurea (Ait.) Benth. (Fabaceae) in Rats" was published in 2022. Journal: Evid Based Complement Alternat Med.

Herbal products are widely utilized by the majority of the population in impoverished nations to alleviate various health problems [5]. According to the world health organization (WHO) report, natural products are used by nearly 80% of the population in Africa due to their affordability, availability, and minimal untoward effects [6, 7]. Almost 25% of modern medicines in drug formulary and many other synthetic equivalents are derived from herbal remedies [8].

*Calpurnia aurea* (Ait.) Benth. (Fabaceae) is a seasonal plant that belongs to the family Fabaceae. The genus comprises short trees that grow in or near woodlands in different regions of Ethiopia. They are also abundant in Africa, ranging from Cape Province to Eritrea, as well as in South India [9]. It has a variety of names in Ethiopia, including “Chekata” (in Oromifa) and “Digita” (in Amharic) [10].

In Ethiopian folkloric medicine, different plant portions are widely employed for numerous human and animal ailments [11]. The leaf segments of the plant are traditionally used to treat several ailments such as syphilis, malaria, rabies, diabetes, hypertension, and diarrhea [12, 13]; whereas the root part of the plant is frequently utilized for amebiasis and giardiasis [14]. In addition, the ethnobotanical survey reported that the leaf part of the plant as a juice is being taken orally for seven days in Gondar Zuria, North West Ethiopia, to heal peptic ulcers [15].

Furthermore, the diverse parts of the plant are experimentally verified to have much therapeutic importance, including antihypertensive [16], antimalarial [17], wound healing, and anti-inflammatory activity [18]; in vitro antibacterial and antioxidant activity [19]; and insecticidal activity [20].

Multiple conventional medicines are available commercially to treat the disease, but they come with many adverse effects, the possibility of relapse on long-term use, and treatment failure [21]. Hence, searching for safe and very effective alternative therapies from natural products is highly demanding. Despite the leaves of the plant is traditionally utilized to relieve gastric ulcer [15], its healing efficacy and safety profile are not yet experimentally authenticated. Thus, the study was carried out to assess the acclaimed ulcer-healing activity and nontoxic profile of the leaf of *Calpurnia aurea* (Ait.) Benth.

The article "Evaluation of the Antiulcer Activity of Methanolic Extract and Solvent Fractions of the Leaves of Calpurnia aurea (Ait.) Benth. (Fabaceae) in Rats" was published in 2022. Journal: Evid Based Complement Alternat Med.

## 2. Materials and Methods

### 2.1. Drugs, Chemicals, and Instruments Used

The following chemical reagents and drugs were employed to carry out the study: absolute ethanol (Blulux Laboratories (P) Ltd., India), phenolphthalein (Blulux laboratories Pvt., India), absolute methanol (AppliChem, Germany), omeprazole (Cadila Pharmaceutical Industries Pvt, India), cimetidine (ACILOC, Cadila, Ethiopia), hydrochloric acid (Blulux Laboratories (P) Ltd., India), ketamine hydrochloride (Neon Laboratories Limited, India), sucralfate (Fourrts Laboratories Pvt., India), normal saline (Cadila Pharmaceuticals, Bengaluru, India), Wagner's reagent (Research-Lab Fine Chem Industries, India), lead acetate 1% (Guangdong Guanghua Chemical Factory, China), ferric chloride (Blulux Laboratories (P) Ltd., India), NaOH (Blulux Laboratories (P) Ltd., India), sulfuric acid (HiMedia Laboratories Pvt. Ltd., India), pH meter (Adwa AD8000), hand lens (10x), centrifuge (Eppendorf AG-5703DQ713856), and lyophilizer (LabFreez Instruments Group Co., Ltd., Japan). All of the supplies were of analytical grade and sourced from the governmental supply agency and other local vendors.

### 2.2. Experimental Animals

Wistar rats (150–200 g) of either sex, which were obtained in the animal house of the School of Pharmacy, University of Gondar, and bought from the Ethiopian Public Health Institute (EPHI), were utilized. They were maintained in individual cages with softwood chips as beddings at 25 ± 2°C on a 12/12-h diurnal cycle.

They were given unlimited access to standard pellet feed and water ad libitum and adapted to the laboratory environment for seven days before initiating the actual experiment.

The experiment was undertaken in compliance with local ethical and internationally accepted regulations for the use, care, and welfare of laboratory animals [22].

### 2.3. Plant Material Collection and Identification

In October 2020, bulk leaves of *Calpurnia aurea* were gathered from Gondar Zuria, 698 km away from the capital city of Ethiopia, Addis Ababa, in the northwest direction. Meanwhile, a small sample of the plant was sent to University of Gondar for verification and identified by a botanist. The given specimens were deposited there in the Department of Biology, the University of Gondar, with registration number (AY002) for future reference.

### 2.4. Preparation of Crude Extract and Fractionation

The bulk leaves of *C. aurea* were washed with cold water and shade dried for 14 days at ambient temperature and then ground into coarse powder using a miller. After that, 600 g of powder was obtained and macerated with a sufficient amount of 80% methanol using a conical flask for 72 h using a mini orbital shaker. On the third day, the supernatant was first isolated from the marc by using gauze twice and then filtered by Whatman No. 1 filter paper. Then, for the second and third time, the remaining residue was re-macerated for six days using a similar solvent. The supernatant from each subsequent filter was mixed and dried under a hot oven set at 40°C, followed by lyophilization to eliminate the moisture. The percentage yield was then computed and maintained in a desiccator with a plastic container [18].

The article "Evaluation of the Antiulcer Activity of Methanolic Extract and Solvent Fractions of the Leaves of Calpurnia aurea (Ait.) Benth. (Fabaceae) in Rats" was published in 2022. Journal: Evid Based Complement Alternat Med.

With minor modification, the hydromethanolic extract was further fractionated by using distilled water, chloroform, and ethyl acetate, as explained by Ayal et al. [18]. Eighty grams of the extract were dissolved in 360 mL distilled water in a separatory funnel and partitioned three times using 360 mL chloroform. To get the chloroform fraction, the precipitate was then condensed in an oven under reduced pressure at 40°C. In the same fashion, the leftover was then partitioned subsequently three times using equal volume of ethyl acetate. The filtrates were then left to dry in a hot oven similar to chloroform fraction. Then, the residual aqueous fraction was lyophilized overnight and the percent yields of individual fractions were determined (in %). Eventually, the products were preserved at −4°C in an airtight container till utilized for experimentation.

### 2.5. Phytochemical Screening Test

For both crude extract and solvent fractions, standard protocols were adopted to conduct phytochemical screening assays for the presence of a wide range of phytochemicals [23, 24].

### 2.6. Acute Oral Toxicity Test

To perform acute toxicity study, the animals were given a limit test dose of 2 g/kg using OECD 425 guidelines. Thus, five female, healthy, and nonpregnant Wistar rats weighing 150–200 g were allocated arbitrarily and housed in an individual cage. After being fasted, a single dose of the test extract (2 g/kg) was administered to a single rat and thus monitored for overt toxicity and fatality for 24 h. Following the effect on the first animal, the next four rats were given a similar dose of the test extract and strictly followed for any peripheral and central anomalies for 14 days [25].

### 2.7. Grouping and Dosing of Animals

Thirty Wistar rats of either sex (150–200 g) were employed and arbitrarily divided into five distinct groups, each with six mice for each model. The negative control was administered distilled water (DW, 10 mL/kg) and assigned to group I; whereas the test extract at 100, 200, and 400 mg/kg were given for group II, III, and IV, respectively; and omeprazole (20 mg/kg), sucralfate (100 mg/kg), and cimetidine (100 mg/kg) were given for positive controls in pyloric ligation-, acidified ethanol-, and acetic acid-induced ulcer models, respectively. In all those models, the groups were assigned as group V. Based on the acute toxicity results, the given doses of the extract were calculated and provided for one week for the first two models and two weeks for the third model.

The article "Evaluation of the Antiulcer Activity of Methanolic Extract and Solvent Fractions of the Leaves of Calpurnia aurea (Ait.) Benth. (Fabaceae) in Rats" was published in 2022. Journal: Evid Based Complement Alternat Med.

To check the antiulcer activity of fractions, the acidified ethanol-induced ulcer model was selected. Sixty-six Wistar rats (150–200 g) of either sex were placed into eleven groups, each with six mice. Negative control groups (group I) was treated with DW (10 mL/kg). Group II, III, and IV were administered 100, 200, and 400 mg/kg chloroform fractions, respectively. Likewise, the ethyl acetate fraction was given in the equivalent doses in ascending order, and the mice were assigned as group V, VI, and VII, respectively; whereas the aqueous fractions at 100, 200, and 400 mg/kg were given for a particular group of mice and they were assigned as group VIII, IX, and X; and the reference drug (sucralfate, 100 mg/kg) was administered for the last group (XI) and it was served as a positive control. All the given doses were provided orally for 7 days.

### 2.8. Pyloric Ligation-Induced Ulcer Model

The investigation was performed using the Shay method with certain modification [26]. The animals were treated as indicated under the Section 2.7. The rats were then forced for starvation for 24 h. One hour after the last treatment, pyloric ligation was performed in all rats to trigger peptic ulcers. The abdomen was then opened by using a minor incision 2 centimeters below the xiphoid process, immobilized using ketamine HCl (75 mg/kg, IP). Then, with care to avoid traction to the pylorus, the pyloric part of the stomach was gently pushed out and ligated. The abdomen was returned with care, and the wall was closed with interrupted suturing with chromic catgut. Following six hours of pyloric ligation, the animals were euthanized by cervical dislocation. The stomach was then isolated, and the contents were poured into the calibrated tube and forced to centrifuge for 10 min at 1000 rpm. Afterward, the purified liquids were then prepared to measure gastric volume, pH, and acidity.

### 2.9. Macroscopic Assessment of the Stomach

The stomach was then dissected along the larger curvature, rinsed in normal saline to dislodge gastric residuals, and viewed under 10x magnifying hand lens to see the formation of ulcers. Using the methods explained by Kulkarni, the total numbers of ulcers were tallied and graded (0 = no ulcer, 0.5 = red coloration, 1 = spot ulcers, 2 = deep ulcers, and 3 = perforations) [27]. After that, the ulcer index (UI) and percent ulcer inhibition (%UI) were articulated using the algorithm below:

(1) $$\begin{array}{c} \text{UI}=\frac{\text{UN}+\text{US}+\text{UP}}{10}, \end{array}$$

where UI = ulcer index; UN = average number of ulcer per animal; US = average severity score, and UP = percentage of animals with ulcer.

(2) $$\begin{array}{c} \%\text{ulcer inhibition}\left(\%\text{UI}\right)=\frac{\text{UI control}-\text{UI pretreated}}{\text{UI control}}\times 100\text{.} \end{array}$$

The article "Evaluation of the Antiulcer Activity of Methanolic Extract and Solvent Fractions of the Leaves of Calpurnia aurea (Ait.) Benth. (Fabaceae) in Rats" was published in 2022. Journal: Evid Based Complement Alternat Med.

### 2.10. Determination of Gastric Volume and pH

The stomach contents were emptied into measuring tubes, centrifuged for 10 min at 1000 rpm, and then the volume of the supernatant was recorded. Then, 1 mL of gastric juice was aliquoted out of the supernatant, mixed with 1 mL of distilled water, and the pH of the solution was determined using a pH meter.

### 2.11. Determination of Total Acidity

After recording the pH, a 50 mL conical flask was filled with a sample of 1 mL gastric juice dissolved with 1 mL of distilled water. After that, 2–3 drops of phenolphthalein were added and titrated with 0.01 N NaOH until a persistent pink color was attained. The quantity of 0.01 N NaOH utilized was noted. The total acidity was then estimated using this formula in mEq/L [28]:

(3) $$\begin{array}{c} \text{Acidity}\left(\text{mEq}/\text{L}\right)=\frac{\text{VNaoH}\times \text{N}\mathrm{\times 100}\;\text{mEq}/\text{L}}{0.1}, \end{array}$$

where *V* = volume and *N* = normality.

### 2.12. Determination of Gastric Mucus Content

The following standard procedure was adopted to determine gastric wall mucus with minor changes [29]. The glandular sections from the stomach were excised and weighed. For 2 h, each section was immersed in 10 mL of 0.1% Alcian blue 8GX solution (in 0.16 M sucrose solution, buffered with 0.05 M sodium acetate, and adjusted to pH 5.8). The residual dye was cleared by washing twice with 0.25 M sucrose solution for 15 and 45 min. The dye chelated with the mucus on the gastric wall was then separated using 20 mL of 0.05 M magnesium chloride with occasional stirring. After that, 5 mL volume of blue extract was shaken for 2 h every 30 min with an equal amount of diethyl ether. Using a UV-visible spectrophotometer at 580 nm, the mixture was then centrifuged for 15 min at 3000 rpm, and the absorbance of the aqueous layer was determined and recorded. The concentration of Alcian blue extracted/g (net) of glandular tissue was then computed using the Alcian blue standard curve.

The article "Evaluation of the Antiulcer Activity of Methanolic Extract and Solvent Fractions of the Leaves of Calpurnia aurea (Ait.) Benth. (Fabaceae) in Rats" was published in 2022. Journal: Evid Based Complement Alternat Med.

### 2.13. Acidified Ethanol-Induced Ulcer Model

In this model, the antiulcer activity of the test extract was assessed using Hara and Okabe's (1985) approach with some modifications [30]. The animals were starved for 24 h and then treated as indicated under the Section 2.7. The animals were given 1 mL/150 g of acidified ethanol solution to induce ulcer after an hour of the last treatment. Following 1 h of induction, the rats were killed by cervical dislocation. The stomachs were removed and carefully cleaned with normal saline. After 10 min, the stomach was then dissected along the anterior surface and observed using 10x hand lens to check the formation of ulcers. The ulcer score, ulcer index (UI), and percent ulcer inhibition were articulated as stated earlier in the pyloric ligation-induced ulcer model.

### 2.14. Acetic Acid-Induced Chronic Ulcer Model

The rats were deprived of food for 24 h and divided arbitrarily into five groups accordingly. After that, they were immobilized using ketamine (75 mg/kg, i.p.) and their stomachs were opened through a midline incision. Acetic acid (20%, 30 *μ*L) was then administered into the subserosal layer with a tiny syringe (0.05 mL). Following 45 seconds of administration of the inducer, the stomach was carefully washed with saline to prevent adhesion to the anterior portion of the ulcerated region and the abdomen was then sealed by employing cat gut no. 2/0. One day after giving the inducer, treatments were given for each group for 2 weeks. On the 15th day, rats were killed, and their stomachs were excised, dissected along the major curvature, and viewed with a 10x magnifying hand lens [31]. Eventually, the ulcer score, ulcer index (UI), and percent ulcer inhibition were computed as indicated in the pyloric ligation method.

### 2.15. Data Analysis

SPSS statistical software, version 24, was used to enter and analyze the data. The values were illustrated as mean ± SEM. Across groups, statistical analysis was performed by employing one-way ANOVA, and comparisons in between groups were carried out using Tukey's post hoc test. When the *P*-value is less than 0.05, the findings were confirmed to be significant.

## 3. Results

### 3.1. Extraction Yields of the Crude Extract and Solvent Fractions

At the end of extraction, 120 g crude extract was harvested (yield = 20%). Eighty grams of the extract was further processed for fractionation from the total product. Afterward, each fraction's yields were calculated and found to be 21.7%, 25%, and 53.3% for chloroform, ethyl acetate, and aqueous fractions, respectively.

### 3.2. Phytochemical Screening Test

Both the crude extract and solvent fractions of the leaf of the plant were screened for phytochemicals and showed the presence of various bioactive principles (Table 1).

The article "Evaluation of the Antiulcer Activity of Methanolic Extract and Solvent Fractions of the Leaves of Calpurnia aurea (Ait.) Benth. (Fabaceae) in Rats" was published in 2022. Journal: Evid Based Complement Alternat Med.

### 3.3. Acute Oral Toxicity Study

During the 14-day follow-up period, the test extract was safe and did not show any lethality following a single limit test dose administration of 2 g/kg. Besides, the crude extract at this dose did not show any delayed overt toxicity such as central and behavioral anomalies.

### 3.4. Effects of the Crude Extract on Pyloric Ligation-Induced Ulcer

In this model, the cytoprotective effect of *C. aurea* leaf extract is illustrated in Table 2. At these respective doses (100, 200, and 400 mg/kg), the extract exhibited a reduction in ulcer index, stomach volume, and overall acidity while raising gastric pH. Relative to the vehicle, among the three respective doses, groups given 200 and 400 mg/kg showed a substantial reduction in ulcer index (*P* < 0.05), the volume of secretion (*P* < 0.05), and total acidity (*P* < 0.05); while, at these doses, gastric pH was raised (*P* < 0.05). In contrast, the effect of the extract at the minimal dose (100 mg/kg) was negligible, which is not statistically significant. It was clearly seen that ulceration was produced after pyloric ligation. However, in groups treated with the leaf extract, gastric ulceration reduced in a dose-dependent manner (Figure 1). The percent ulcer reduction was reported to be 3.3%, 37.1%, and 54% in groups treated with 100, 200, and 400 mg/kg doses, respectively. The administration of the maximum dose (400 mg/kg) of the test extract resulted in the greatest reduction in ulcer index (54%), which is comparable to the existing drug (55.4%).

### 3.5. Effects of the Crude Extract on Gastric Mucus Content

The activity of the test extract on stomach mucus content was examined by using the pyloric ligation-induced ulcer method. In comparison with the vehicle, the findings confirmed that the stomach mucin level was significantly enhanced in groups that received the test extract at 200 (*P* < 0.05) and 400 mg/kg (*P* < 0.001). In groups that received distilled water (negative controls), the mean mucus content was reported to be 61.64 ± 1.05 *μ*g/g. However, in groups that received the test extract at both test doses, the mean stomach mucus content was dramatically raised to 67.46 ± 1.00 and 74.77 ± 1.53 *μ*g/g, respectively. Furthermore, at 100 mg/kg, the impact on gastric mucin content was assessed and found to be 63.84 ± 1.3 *μ*g/g, which is negligible (*P* > 0.05). At the ceiling dose of the test extract (400 mg/kg), the peak gastric mucin level was attained, which is nearly equivalent to the reference drug (Table 2).

The article "Evaluation of the Antiulcer Activity of Methanolic Extract and Solvent Fractions of the Leaves of Calpurnia aurea (Ait.) Benth. (Fabaceae) in Rats" was published in 2022. Journal: Evid Based Complement Alternat Med.

### 3.6. Effects of the Crude Extract on Acidified Ethanol-Induced Ulcer

In groups given the vehicle (DW), the inducer causes considerable ulcer formation, with an ulcer index of 17.88 ± 0.23. Nonetheless, when compared with the negative control, groups of rats given the extract at doses of 200 (*P* < 0.01) and 400 mg/kg (*P* < 0.001) considerably lowered the ulcer index (Figure 2). For both doses, the ulcer index was dropped to 12.96 ± 0.30 and 10.32 ± 0.09, respectively. In groups of rats administered 100 mg/kg of the test extract, however, the reduction in ulcer index was minimal and statistically insignificant. In this model, the activity of the test extract was proved to be dose-dependent. The cytoprotective effect was evaluated through percent ulcer inhibition and was reported to be 5.6%, 27.5%, and 42.3% for 100, 200, and 400 mg/kg test doses, respectively; whereas, in groups of rats given the reference drug (sucralfate), the percent ulcer inhibition was 44.8%, which is comparable to the test extract at the highest dose (42.3%). The findings revealed that the crude extract had a substantial cytoprotective effect at both doses (200 and 400 mg/kg), while the activity at 100 mg/kg was negligible (Table 3).

### 3.7. Effects of the Crude Extract on Acetic Acid-Induced Ulcer

After 14 days of treatment, the leaf extract of the plant at both test doses (200 and 400 mg/kg) dramatically healed the ulcer (*P* < 0.001). At these respective doses, the ulcer-healing effect was assessed by computing percent ulcer reduction and was found to be 53.22% and 54.59%, respectively. In contrast, relative to the negative control, the plant extract at 100 mg/kg displayed comparatively minimal ulcer reduction (*P* > 0.05); whereas the ulcer-healing activity of the test extract at 200 and 400 mg/kg was statistically significant and demonstrated a considerable reduction in ulcer index (*P* < 0.001). The maximal ulcer-healing activity of the test extract was observed at 400 mg/kg (53.6%), which is nearly equivalent to the reference drug (54.2%). The findings are shown in Table 4 and Figure 3.

### 3.8. Effects of the Solvent Fractions on Acidified Ethanol-Induced Ulcer

Following the crude extract evaluated using the previous three models, the cytoprotective effect of each solvent fraction was further examined by utilizing the acidified ethanol-induced ulcer method. At all test doses, groups of rats given ethyl acetate fraction showed statistically significant reduction (*P* < 0.05) on ulcer index in a dose-dependent manner.

Correspondingly, the cytoprotective effect of the aqueous fraction was also examined and was found to be significant at 400 mg/kg (*P* < 0.001). On the contrary, relative to that of the vehicle, the aqueous fractions at the rest doses did not show considerable ulcer index variation (Figure 4). In addition, at the given doses, the effect of chloroform fraction was assessed, and it could not lower ulcer index appreciably (*P* > 0.05). In groups given ethyl acetate fraction, the percent ulcer inhibition was increased in a dose-dependent manner and was found to be 14.2%, 25.6%, and 52.4%, respectively. At the three respective doses, an aqueous fraction reduced the ulcer index by 4.2%, 5.0%, and 41.5%, respectively.

The article "Evaluation of the Antiulcer Activity of Methanolic Extract and Solvent Fractions of the Leaves of Calpurnia aurea (Ait.) Benth. (Fabaceae) in Rats" was published in 2022. Journal: Evid Based Complement Alternat Med.

Overall, when compared with the vehicle, the ethyl acetate fraction at all test doses and aqueous fraction at ceiling doses (400 mg/kg) were capable to reduce the ulcer index significantly. The ethyl acetate fraction at 400 mg/kg offered the best ulcer prevention when compared with all other fractions (52.4%). In depth, the findings are summarized in Table 5 and Figure 5.

## 4. Discussion

Even though the causes of peptic ulcers are not known clearly, it has been scientifically proven that they are caused by an imbalance between offensive and defensive elements [32]. Despite the fact that numerous modern medicines are accessible for healing peptic ulcers, the majority of these pharmaceuticals have serious side effects. Herbal remedies are the basis for new potential candidates, and they have been established to be beneficial in combating both gastric and duodenal ulcers [33].

To validate the ulcer-healing potential and probable mechanisms of the hydromethanolic extract of *Calpurnia aurea* leaves, the investigators employed three distinct ulcer models, including acidified ethanol-, pyloric ligation-, and acetic acid-induced gastric ulcer methods. These three scientific models were chosen because they best meet the aims of evaluating antisecretory and gastroprotective properties of the test extract.

In the study, the quantity of the crude extract after extraction was measured and was found to be 20% (120 g), which is consistent with the earlier findings [18]. During extraction, hydromethanolic solvents were used since the co-solvents are well studied and thought to give adequate products, and a wide range of secondary metabolites owing to their good polarity index [34].

The acute toxicity study indicated that the crude extract showed no evidence of any noticeable manifestations of delayed toxicity during the strict 14-day follow-up period. In addition, no death was noticed at the limited test dose, which is 5 times the maximal dose of the test extract (400 mg/kg). If the extract's lethal dose (LD50) is greater than three times the minimum effective dose, it could be a potential candidate for future research [35]. As a result, lack of detection of death at 2 g/kg demonstrated that the plant leaf extract is nontoxic and its LD50 is likely to be far from the limit test dose.

The article "Evaluation of the Antiulcer Activity of Methanolic Extract and Solvent Fractions of the Leaves of Calpurnia aurea (Ait.) Benth. (Fabaceae) in Rats" was published in 2022. Journal: Evid Based Complement Alternat Med.

Using a pyloric ligation-induced ulcer method, the gastroprotective potential of the leaves of the hydromethanolic extract was investigated. The method was chosen because it resembles some of the most common stomach ulcers in humans. Following pyloric ligation, it is well investigated that there will be acid-pepsin deposition, resulting in mucosal digestion. Consequently, the production of prostaglandin E2 and I2, which are regulators for suppressing stomach acid secretion, increasing mucus, and bicarbonate formation, is reduced [36]. An additional scientific study revealed that a disruption in gastric blood circulation and an increase in oxidative stress might be accountable for ulcer formation [26, 37]. The model was adopted to analyze the antisecretory and gastroprotective effects of the promising agent.

In this model, following administering the crude extract at 200 and 400 mg/kg doses, there was a marked decline (*P* < 0.01) in ulcer index, the volume of stomach acid, and overall acidity. Moreover, at a similar dose, the impact of the crude extract was examined in terms of stomach pH and gastric mucus content and was found to be statistically significant. Nonetheless, the activity of the test extract at 100 mg/kg in the given parameters was negligible (*P* > 0.05). This implied that the lowest dose of the extract is insufficient to provide cytoprotective and antisecretory properties. The discrepancy in activity could be attributed to the absence of an adequate concentration of active phytochemical constituents. Consequently, the investigations demonstrated that at medium and higher doses, the hydromethanolic extract had excellent gastroprotective and antisecretory effects. Overall, the finding supported that the plant extract showed remarkable antiulcer activity, owing to cytoprotective and antisecretory properties.

As identified by phytochemical assay, the hydromethanolic extract comprised a broad range of bioactive ingredients, such as flavonoids, tannins, and saponins. Numerous scientific studies showed that flavonoids have been scientifically proven to have gastroprotective and antisecretory effects [38]. Likewise, phenolic substances and flavonoids enhance capillary resistance and improve microcirculation by generating prostaglandin and antioxidant enzymes [39, 40]. Tannins shield the outermost layer of the mucosa and remodel its structure, making it more resistant to dangerous toxic agents [41]. Saponins and triterpenoids are reported to have the ability to produce mucus [36]. As a result, the crude extract's considerable antiulcer activity and excessive mucus production could be linked to the presence of such bioactive ingredients.

The article "Evaluation of the Antiulcer Activity of Methanolic Extract and Solvent Fractions of the Leaves of Calpurnia aurea (Ait.) Benth. (Fabaceae) in Rats" was published in 2022. Journal: Evid Based Complement Alternat Med.

Using an acidified ethanol-induced gastric ulcer method, the ulcer-relieving potential of the hydromethanolic extract of *Calpurnia aurea* leaves was also explored. The approach was chosen since it is identical to what has been found in human cases of excessive acid production. The model was applied to determine the test extract's cytoprotective properties. In this model, HCL was used to hasten the ulcerogenesis pathway, exacerbate lesions, and diminish the mucosal protection against toxic substances [30].

Following induction with acidified ethanol, the ulcer index was found to be high in negative controls. However, in tested groups pretreated with 200 and 400 mg/kg extract, the values of ulcer index dropped dramatically. The effect of the plant extract at the dose of 100 mg/kg, on the other hand, was observed to be minimal (*P* > 0.05). Therefore, it is possible to conclude that the hydromethanolic extract at the lowest dose exhibited no ulcer-healing activity.

In the experimental procedure, ethanol is frequently utilized to trigger ulcers in laboratory animals, causing extensive gastrointestinal mucosa lesions. Studies demonstrated that injury to the gastric mucosa is thought to begin with vascular endothelial disruption, causing enhanced vascular permeability, edema, and epithelial lifting [42]. In addition, because of its direct toxic action, ethanol causes intensive injury in the gastrointestinal mucosa, diminishing bicarbonate and mucus production [43].

The study findings revealed that the plant extract at medium and higher doses showed substantial cytoprotective activity. The boost in mucosal prostaglandin concentration elicited by the test extract, owing to flavonoids, could be the possible mechanism for the observed effect [44]. Similarly, additional bioactive compounds such as tannins may contribute to the desired ulcer-healing activity. Indeed, bioactive ingredients like tannins are among the gastroprotective active compounds in which antiulcer activity has been intensively explored [45].

Acidified ethanol would severely injure the gastrointestinal mucosa, resulting in enhanced neutrophil migration and liberation of pro-inflammatory mediators and free radicals. It has been shown that suppressing neutrophil migration during inflammation could help to relieve peptic ulcers [46]. Thus, the hydromethanolic extract's antiulcer activity could be associated with the existence of flavonoids, which have been widely investigated for their anti-inflammatory effect [47]. Studies have also reported that the plant's leaf had both *in vitro* and *in vivo* anti-inflammatory activity [18, 48]. Hence, it is possible to conclude that the action of the plant extract can be related to its anti-inflammatory properties. The findings are in concordance with the earlier study, which proved that the gastroprotective potential of curcumin extract is linked to its anti-inflammatory activity [49].

The article "Evaluation of the Antiulcer Activity of Methanolic Extract and Solvent Fractions of the Leaves of Calpurnia aurea (Ait.) Benth. (Fabaceae) in Rats" was published in 2022. Journal: Evid Based Complement Alternat Med.

Acidified ethanol could also induce gastric mucosal injury probably through generation of leukotrienes and activation of 5-lipoxygenase pathway. Leukotriene antagonists and 5-lipoxygenase blockers have been shown to prevent ethanol-induced stomach ulcers [33]. As a result, the cytoprotective effects of *Calpurnia aurea* leaf extract might be related to blocking the 5-lipoxygenase pathway or leukotriene activity.

Antioxidants have been shown to safeguard the gastrointestinal mucosa from oxidative damage caused by ethanol [50]. There was also a scientific study that providing antioxidants is significant to warrant gastric ulcers due to ethanol [51]. Interestingly, in prior investigations, *Calpurnia aurea* leaf extract has been proven to have *in vitro* antioxidant activity [11]. Therefore, it is plausible that this plant's gastroprotective properties could be accredited to its antioxidant potential.

By adopting the acetic acid-induced chronic ulcer method, the ulcer-healing potential of the plant extract was also explored. The model causes severe, difficult to heal ulcer in the stomach wall, analogous to chronic ulcers in human beings [52]. It has been known that the inducer causes gastric ulcers by obstructing the gastrointestinal mucosa, resulting in a massive concentration of acidic gastric juice [53]. In this model, following 14 days of treatment, the plant extract significantly lowered the ulcer index (*P* < 0.001) at both test doses (200 and 400 mg/kg).

It is well documented that gastroprotective action alone in rodents does not cause tremendous antiulcer activity in human beings. Consequently, the ulcer-relieving activity of the hydromethanolic extract in humans could be related to both antisecretory and cytoprotective properties. The antiulcer effect could be attributed to flavonoids, which have been shown to have an antioxidant effect. Flavonoids are also implicated in augmenting the release of prostaglandins, thereby stimulates crucial mucosal-protecting factors [44]. Moreover, the antiulcerogenic action might be connected to the renewal of blood vessels by saponins via improved VEGF expression [54]. Hence, the plant extract's antioxidant and angiogenesis properties might be beneficial in resolving ulcers.

The article "Evaluation of the Antiulcer Activity of Methanolic Extract and Solvent Fractions of the Leaves of Calpurnia aurea (Ait.) Benth. (Fabaceae) in Rats" was published in 2022. Journal: Evid Based Complement Alternat Med.

In the study, by employing the acidified ethanol-induced ulcer method, the antiulcer effect of each fraction was also assessed in rats. All the given doses of the ethyl acetate fraction had shown substantial gastroprotective activity, which is in consonance with the recent study conducted in *Rumex nepalensis* root extract [54]. Comparably, at the maximal dose (400 mg/kg), the antiulcer activity of the aqueous fraction was also found to be substantial. In contrast, no notable antiulcer activity has been observed in any doses of the chloroform fraction. As per phytochemical screening assay, chloroform fraction was free of saponins, flavonoids, terpenoids, tannins, and phenols. The ethyl acetate and aqueous fractions, on the other hand, were plentiful in the aforementioned bioactive molecules. Hence, it is conceivable that these are the factors why the ethyl acetate and aqueous fractions of *C. aurea* have exhibited considerable antiulcer activity.

## 5. Conclusions

The study demonstrated that the hydromethanolic extract and solvent fractions were shown to have excellent antiulcer activity. The observed antiulcer potential could have been attributed to the existence of diverse bioactive molecules in the plant. The precise mode of action of extracts is unknown, but antisecretory and cytoprotective activities may indeed be responsible for the required ulcer-healing effect.

## Figures and Tables

**Figure 1:** Effects of crude extract of *C. aurea* in pyloric ligation-induced ulcer rats: (a) groups given distilled water (10 mL/kg), (b) groups given 100 mg/kg test extract, (c) groups given 200 mg/kg test extract, (d) groups given 400 mg/kg test extract, and (e) groups given the reference drug (omeprazole 20 mg/kg).

**Figure 2:** Effects of crude extract of *C. aurea* in acidified ethanol-induced ulcer rats: (a) groups given distilled water (10 mL/kg), (b) groups given 100 mg/kg test extract, (c) groups given 200 mg/kg test extract, (d) groups given 400 mg/kg test extract, and (e) groups given the reference drug (sucralfate 100 mg/kg).

**Figure 3:** Effects of crude extract of *C. aurea* in acetic acid-induced ulcer rats: (a) groups given distilled water (10 mL/kg), (b) groups given 100 mg/kg test extract, (c) groups given 200 mg/kg test extract, (d) groups given 400 mg/kg test extract, and (e) groups given the reference drug (cimetidine 100 mg/kg).

**Figure 4:** Effects of solvent fractions of *C. aurea* in acidified ethanol-induced ulcer rats: (a) groups given distilled water (10 mL/kg), (b) groups given 100 mg/kg CF, (c) groups given 200 mg/kg CF, (d) groups given 400 mg/kg CF, (e) groups given 100 mg/kg AF, (f) groups given 200 mg/kg AF, (g) groups given 400 mg/kg AF, (h) groups given 100 mg/kg EF, (i) groups given 200 mg/kg EF, (j) groups given 400 mg/kg EF, and (k) groups given sucralfate 100 mg/kg.

The article "Evaluation of the Antiulcer Activity of Methanolic Extract and Solvent Fractions of the Leaves of Calpurnia aurea (Ait.) Benth. (Fabaceae) in Rats" was published in 2022. Journal: Evid Based Complement Alternat Med.

**Figure 5:** Percent ulcer inhibition of solvent fractions of *C. aurea* leaf extract in acidified ethanol-induced ulcer rats.

**Table 1:** Phytochemical screening of the leaf of *Calpurnia aurea* crude extract and solvent fractions.

Secondary metabolites	Tests utilized for screening	Crude extract	Chloroform fraction	Ethyl acetate fraction	Aqueous fraction
Alkaloids	Wagner's test	+	−	+	−
Tannins	Ferric chloride test	+	−	+	+
Terpenoids	Salkowski's test	+	−	+	+
Flavonoids	Lead acetate test	+	−	+	+
Saponins	Foam test	+	−	+	+
Phenols	Sodium hydroxide test	+	−	+	+
Steroids	Salkowski's test	+	+	−	−
Glycosides	Glycoside test	+	+	+	+
Anthraquinones	Borntrager's test	−	−	−	−

Note: (+): present, (−): absent.

**Table 2:** The impact of *Calpurnia aurea* crude extract on ulcer index, gastric volume, total acidity, pH, and stomach mucin level in pyloric-ligated rats.

Group	Ulcer index	%UI	Gastric volume (mL)	pH	Acidity in mEq/L	Mucus content (*μ*g/g)
NC	17.75 ± 1.82	—	2.97 ± 0.46	2.08 ± 0.05	51.65 ± 1.42	61.64 ± 1.05
CALE100	17.17 ± 1.39	3.3	2.83 ± 0.44	2.32 ± 0.08	50.16 ± 2.15	63.84 ± 1.31
CALE200	11.17 ± 2.39e^*∗∗*^	37.1	2.80 ± 0.24	2.73 ± 0.20e^*∗∗*^	47.53 ± 0.76e^*∗*^	67.46 ± 1.00e^*∗*^
CALE400	8.17 ± 2.60e^*∗∗∗*^	54	1.32 ± 0.10e^*∗∗∗*^	4.73 ± 0.05e^*∗∗∗*^	32.81 ± 0.45e^*∗∗∗*^	74.77 ± 1.53e^*∗∗∗*^
OM20	7.92 ± 2.51e^*∗∗∗*^	55.4	1.28 ± 0.10e^*∗∗∗*^	4.88 ± 0.09e^*∗∗∗*^	31.27 ± 0.61e^*∗∗∗*^	78.50 ± 1.10e^*∗∗∗*^

Values are expressed as mean ± SEM (*n* = 6) and analyzed using one-way ANOVA, followed by Tukey's post hoc test. ^e^Compared with negative control. ^*∗*^*P* < 0.05, ^*∗∗*^*P* < 0.01, and ^*∗∗∗*^*P* < 0.001. NC = negative control, CALE = *Calpurnia aurea* leaf extract, OM20 = omeprazole 20 mg/kg, %UI = percent ulcer inhibition, mL = milliliter, mEq/*L* = milliequivalents per liter, and *μ*g/g = microgram per gram.

**Table 3:** The effect of *Calpurnia aurea* crude extract on ulcer number, ulcer score, and ulcer index in acidified ethanol-induced ulcer rats.

Group	Mean ulcer number (UN)	Mean ulcer score (US)	Mean ulcer index (UI)	%UI
NC	29.83 ± 1.25	49.00 ± 1.17	17.88 ± 0.23	—
CALE100	26.83 ± 1.78	42.10 ± 3.78	16.87 ± 0.56	5.6
CALE200	12.83 ± 1.17	16.75 ± 1.86	12.96 ± 0.30e^*∗∗*^	27.5
CALE400	1.50 ± 0.22	1.67 ± 0.69	10.32 ± 0.09e^*∗∗∗*^	42.3
SUC100	1.33 ± 0.21	0.83 ± 0.17	9.87 ± 0.04e^*∗∗∗*^	44.8

Values are expressed as mean ± SEM (*n* = 6) and analyzed using one-way ANOVA followed by Tukey's post hoc test. ^e^Compared with negative control. ^*∗∗*^*P* < 0.01, and ^*∗∗∗*^*P* < 0.001. NC = negative control, CALE = *Calpurnia aurea* leaf extract, SUC100 = sucralfate 100 mg/kg, UN = ulcer number, US = ulcer score, UI = ulcer index, and %UI = percent ulcer inhibition.

The article "Evaluation of the Antiulcer Activity of Methanolic Extract and Solvent Fractions of the Leaves of Calpurnia aurea (Ait.) Benth. (Fabaceae) in Rats" was published in 2022. Journal: Evid Based Complement Alternat Med.

**Table 4:** The ulcer-healing effect of *Calpurnia aurea* crude extract on ulcer number, ulcer score, and ulcer index in acetic acid-induced ulcer rats.

Group	Mean ulcer number (UN)	Mean ulcer score (US)	Mean ulcer index (UI)	%UI
NC	36.17 ± 0.87	64.92 ± 1.98	20.11 ± 1.69	—
CALE100	35.67 ± 0.67	55.58 ± 1.58	19.13 ± 1.69	4.9%
CALE200	5.67 ± 0.92	10.50 ± 1.76	11.62 ± 1.69e^*∗∗∗*^	42.2%
CALE400	4.00 ± 0.93	6.00 ± 1.49	9.33 ± 1.69e^*∗∗∗*^	53.6%
CM100	3.67 ± 0.88	5.25 ± 1.56	9.22 ± 1.69e^*∗∗∗*^	54.2%

Values are expressed as mean ± SEM (*n* = 6) and analyzed using one-way ANOVA followed by Tukey's post hoc test. ^e^Compared with negative control. ^*∗∗∗*^*P* < 0.001. NC = negative control, CALE = *Calpurnia aurea* leaf extract, CM100 = cimetidine 100 mg/kg, UN = ulcer number, US = ulcer score, UI = ulcer index, and %UI = percent ulcer inhibition.

**Table 5:** Effects of the solvent fractions of *C. aurea* leaf extract on ulcer number, ulcer score, and ulcer index in acidified ethanol-induced ulcer rats.

Group	Mean ulcer number (UN)	Mean ulcer score (US)	Mean ulcer index (UI)	%UI
NC	69.50 ± 2.75	104.83 ± 4.57	27.43 ± 0.73	—
CF100	68.00 ± 1.91	103.50 ± 2.58	27.15 ± 0.45	1.1
CF200	62.33 ± 1.89	96.00 ± 2.82	25.83 ± 0.47	5.8
CF400	60.83 ± 1.80	90.00 ± 2.45	25.08 ± 0.42	8.6
EF100	53.17 ± 4.21	82.25 ± 6.67	23.54 ± 1.09e^*∗*^	14.2
EF200	41.17 ± 0.60	62.83 ± 1.51	20.40 ± 0.20e^*∗∗∗*^	25.6
EF400	13.67 ± 1.31	17.00 ± 2.25	13.07 ± 0.35e^*∗∗∗*^	52.4
AF100	65.00 ± 1.21	97.67 ± 1.58	26.27 ± 0.27	4.2
AF200	63.33 ± 1.28	97.33 ± 1.97	26.07 ± 0.32	5.0
AF400	26.17 ± 1.08	34.25 ± 1.53	16.04 ± 0.26e^*∗∗∗*^	41.5
SUC100	7.17 ± 0.95	7.92 ± 1.15	11.51 ± 0.21e^*∗∗∗*^	58.0

Values are expressed as mean ± SEM (*n* = 6) and analyzed using one-way ANOVA followed by Tukey's post hoc test. ^e^Compared with negative control. ^*∗*^*P* < 0.05, ^*∗∗*^*P* < 0.01, and ^*∗∗∗*^*P* < 0.001. NC = negative control, CF = chloroform fraction, EF = ethyl acetate fraction, AF = aqueous fraction, SUC100 = sucralfate 100 mg/kg, UN = ulcer number, US = ulcer score, UI = ulcer index, and %UI = percent ulcer inhibition.

## Data Availability

The data sets used in this study are available upon reasonable request from the corresponding author.

## Abbreviations

CA: *Calpurnia aurea*
CF: Chloroform fraction
AF: Aqueous fraction
EF: Ethyl acetate fraction
UI: Ulcer index
LD50: Median lethal dose
NC: Negative control
OECD: Organization for Economic Cooperation and Development
SEM: Standard error of mean
SUC: Sucralfate
VEGF: Vascular endothelial growth factor.
